The article "Clinical Analysis of the Renal Protective Effect of GLP-1 on Diabetic Patients Based on Edge Detection" was published in 2022. Journal: J Healthc Eng.

# Clinical Analysis of the Renal Protective Effect of GLP-1 on Diabetic Patients Based on Edge Detection

**DOI:** 10.1155/2022/6504006

**Published:** 2022-03-22

**Authors:** Jing Wang, Yang Wang, Ping Pang, Xiaomeng Jia, Xu Yan, Zhaohui Lv

**Affiliations:** ^1^Department of Clinical Nutrition, The 8th Medical Center of Chinese PLA General Hospital, Beijing 100091, China; ^2^Department of Nephrology, The 8th Medical Center of Chinese PLA General Hospital, Beijing 100091, China; ^3^Department of Endocrinology, Hainan Branch of Chinese PLA General Hospital, Sanya 572013, China; ^4^Center for Endocrine Metabolism and Immune Disease, Beijing Luhe Hospital, Capital Medical University, Beijing 101149, China; ^5^Department of Endocrinology, The 1st Medical Center of Chinese PLA General Hospital, Beijing 100853, China

## Abstract

With the rapid development of IoT technology, it is a new trend to combine edge computing with smart medicine in order to better develop modern medicine, avoid the crisis of information “sibling,” and meet the requirements of timeliness and computational performance of the massive data generated by edge devices. However, edge computing is somewhat open and prone to security risks, so the security and privacy protection of edge computing systems for smart healthcare is receiving increasing attention. The two groups were compared before and after treatment for blood glucose, blood lipids, blood pressure, renal function, serum advanced glycosylation end products (AGEs) and cyclic adenosine monophosphate (cAMP), serum oxidative stress indicators, and levels of cAMP/PKA signalling pathway-related proteins in peripheral blood mononuclear cells. The results of this study show that the reduction of AGEs, the improvement of oxidative stress, and the regulation of the cAMP/PKA signalling pathway may be associated with a protective effect against early DKD. By introducing the edge computing system and its architecture for smart healthcare, we describe the security risks encountered by smart healthcare in edge computing, introduce the solutions proposed by some scholars to address the security risks, and finally summarize the security protection framework and discuss the specific solutions for security and privacy protection under this framework, which will provide some help for the credible research of smart healthcare edge computing.

## 1. Introduction

As the disease progresses, there are disturbances in glucose metabolism and lipid metabolism in the body, leading to metabolic syndrome characterized by metabolic disorders in patients with diabetes [1, 2]. GHb and lipid metabolism levels can help determine the progression of diabetes and the development of metabolic syndrome in patients. In the present study, waist circumference, BMI, systolic blood pressure, diastolic blood pressure, FBG, GHb, TC, TG, HDL-C, and TNF-*α* values were greater and GLP-1 expression levels were lower in patients with diabetes mellitus combined with metabolic syndrome. The results of this study suggest that several indicators are abnormal in patients with diabetes mellitus combined with metabolic syndrome, and the detection of these indicators can help predict and evaluate the disease process of patients and provide refined data for precise treatment [3]. GLP-1 is intestinal proinsulin, usually produced by intestinal endocrine L cells, mainly from the jejunum, ileum, and colon and is important for the regulation of insulin secretion and release [4]. While inhibiting glucagon levels, it suppresses gastric emptying and promotes satiety, inhibiting feeding [5]. GLP-1 improves insulin sensitivity, increases glucose uptake and utilization, and protects the cardiovascular system [6]. GLP-1 activity and levels in vivo are low due to degradation by dipeptidyl peptidase [7, 8].

The article "Clinical Analysis of the Renal Protective Effect of GLP-1 on Diabetic Patients Based on Edge Detection" was published in 2022. Journal: J Healthc Eng.

In recent years, the inflammatory response has been recognized as one of the causes of diabetes mellitus and the pathogenesis of type 2 diabetes mellitus [9]. TNF-*α*, as the most common and important inflammatory factor, is a common indicator of metabolic syndrome [10]. TNF-*α* not only causes local tissue and systemic inflammatory responses but also contributes to insulin resistance [11]. As the trend towards the Internet of everything continues to deepen, it is helping to move smart healthcare [12] from clinical business informatics to personalised medicine. Smart Healthcare is a patient-centric information system that uses benefits all components of the healthcare ecosystem [13]. As healthcare data continue to accumulate and databases grow, the number of devices on the digital capture, processing, storage, transmission, and decision-making end of healthcare information continues to increase, making the growth of data far faster than the growth of network bandwidth. A report by the International Data Corporation (IDC) states that 50% of IoT networks face network bandwidth limitations by the end of 2018 [14]. At the same time, Cisco reports that IoT devices will also grow rapidly, with 50 billion devices expected to connect to the Internet and generate 600 ZB of data in 2020, with complex network environments placing higher demands on transmission and compute latency. IDC's report [15] also predicts that by 2020 more than 40% of USD trillion. Therefore, it is becoming increasingly important to integrate IoT with cloud computing [16]. Mobile devices utilizing cloud services will lead to latency and mobility-related problems [17], therefore, combining edge computing [18] with smart healthcare is a new trend for new healthcare in a new era [19], where the three common edge computing models are cloudlets [20], fog computing (fog computing) [21], and mobile edge computing (MEC) [22].

The article "Clinical Analysis of the Renal Protective Effect of GLP-1 on Diabetic Patients Based on Edge Detection" was published in 2022. Journal: J Healthc Eng.

Then, it will become promine [23]. According to a report published by Forbes in 2015, cloud-based security spending is expected to increase by 42%; according to another study, IT security spending has increased to 79.1% by 2015, an annual increase of more than 10%. IDC showed in 2011 that 74.6% of enterprise customers cited security as a major challenge. At the same time, smart healthcare is subject to information security risks such as low data quality, leakage of sensitive data, and malicious external theft [24]. To date, there is no unified security protection standard for trusted edge computing for smart healthcare. Therefore, it is urgent to study how to build an effective information security strategy and security operation system for the development of smart healthcare under edge computing.

## 2. Proposed Method

Edge computing is characterized by decentralization, data localization, and low latency [25], and the combination of intelligent healthcare and edge computing is of great significance. On the one hand, it can provide more efficient and convenient medical services and simplify the medical process; on the other hand, it can provide a fairer and more open supply of medical resources, and the information technology on the basis of digitalization will break the “silo” state of medical digital information and form interconnection. A common edge computing architecture for smart healthcare is shown in Figure 1.

The intelligent sensing layer consists of medical sensing devices and data collection devices, which are responsible for the sensing and collection of medical data. The data transmission layer transmits the data collected by the smart perception layer through mobile communication networks, the Internet, and wireless mesh networks.

The data integration layer establishes an integrated innovation system and a model dynamic data center by means of sensing, correlation, and traceability and completes the establishment of an empirical model database and an evidence-based model database according to the different categories of data. The empirical models refer to some key symptoms that cannot be obtained by physical and chemical equipment testing, such as past medical history, family medical history, occupation, external temperature, and season. They also include some incidental indicators, such as low fever in the afternoon, morning cough, irregular menstruation, chest tightness, shortness of breath, vocal changes, small abdominal cramps, dizziness, and dizziness.

The article "Clinical Analysis of the Renal Protective Effect of GLP-1 on Diabetic Patients Based on Edge Detection" was published in 2022. Journal: J Healthc Eng.

The cloud computing layer takes the integrated data transmitted by the data transfer layer and processes it through intensive computing into the functions required by the doctor. Examples include neuronal algorithms, artificial intelligence [26], machine learning, big data processing, symptom trees, and algorithm integration platforms used to process user data.

The application layer is a process that combines certain needs of the healthcare industry to achieve intelligence and is mainly used to address issues such as information processing and human-computer interaction. For example, mobile phone clients: for online users, disease screening portals are designed for patients who have initial knowledge of their own disease to further understand the possibility of that disease. It also effectively enhances the patient consultation experience and reduces patient waiting time in line. After registration, the patient will be given the appropriate physical and chemical indexes through the diagnostic recommendations of the CDSS, and the patient can take the physical and chemical indexes data to complete the doctor's diagnosis and prescription, saving 1/3 of the patient's consultation time and reducing the doctor's workload by 30%.

## 3. Edge Computing Security for Smart Healthcare

Privacy protection issues the combination of smart healthcare and edge computing as an emerging healthcare model has, to a certain extent, enabled the sharing of healthcare information and become an enabler of healthcare reform, providing equal healthcare funding and more accurate healthcare services to patients in all regions. However, as an emerging healthcare model, the openness of edge computing, the diverse data types, and the massive data scale all bring issues such as data security and private security to the edge computing system of smart healthcare. The issue of private security arises from the development of the Internet of Things, awareness of patient rights and interests, and value-added data, as shown in Figure 2.

To better protect the privacy and security of medical data, many experts and scholars have conducted research. Scheen [27] proposed an outsourced cloud data privacy protection scheme for mobile devices, which use probabilistic public key encryption and keyword ranking search algorithms to achieve privacy-preserving ranking queries on resource-constrained mobile terminals. Firstly, the mobile user generates an index of files and encrypts the data and index for upload. Secondly, to access the ciphertext data stored in the cloud. The user generates trapdoors for the keywords and sends them to the cloud. Eventually, the cloud server returns ranked matching data based on relevance score to the user based on the search trapdoors, which in turn decrypts the original data. A location privacy sharing system, MobiShare, was designed in an online mobile social networking environment that enables location sharing between trusted and untrusting users and supports range queries and user-defined access controls. By storing the user's identity and anonymous location information in two separate entities during the sharing process, the user's location privacy can be protected even if one of the entities is attacked.

The article "Clinical Analysis of the Renal Protective Effect of GLP-1 on Diabetic Patients Based on Edge Detection" was published in 2022. Journal: J Healthc Eng.

From the abovementioned references, it can be concluded that the core of protecting user privacy is in 4 areas: data security, privacy protection, authentication, and access control, and its core framework for protecting user privacy is shown in Figure 3.

From the anonymous authentication scheme proposed in [28], it is known that the fundamental goal of anonymously patient-identifiable information is to make it impossible for an attacker to associate user information (sensory data, command information, etc.) with the owner of the information. Therefore, the most intuitive measure of the strength of an algorithm's privacy protection is the information identification rate (IR). The identification rate can generally be obtained statistically but for a given moment the requests in the anonymity region *Q*.

A privacy metric g(q) needs to be given directly, without statistics, such that the set of requests with a larger value of g(q) has a smaller (statistically significant) rate of corresponding information being identified. It is easy to see that there is more than one privacy metric available, and this paper argues that a good privacy metric should satisfy the following relation, i.e., if for a set of requests *Q*={*q|g*(*q*)=*g*_0_} with g(q) value *g*_0_, there exists a theoretical lower bound IR_min_(*g*_0_) on the trajectory recognition rate, then, the closer the actual information recognition rate IR_min_(*q*) is to IR_min_(*g*_0_) the better.

The basic idea is that for a given service request from user *u*_*i*_, *q* is assumed to be protected by *k* anonymity, resulting in an anonymous set of messages for *q*. *U*={*u*_1_, ⋯, *u*_*k*_}. If the probability that user *u*_*i*_ sends *q* is $p\left(u_{i}\overset{\text{cm}}{⟶}q\right)$, then, the entropy of the message “ sender of request q” is $H\left(q\right)=-\sum_{u_{i}\in U}p\left(u_{i}\overset{\text{cm}}{⟶}q\right)\mathrm{lb}p\left(u_{i}{}^{\text{cm}}qq\right)$ according to Shannon's formula. Using the monotonicity of the exponential function, the privacy measure PD(*q*)=2^*H*(*q*)^ can be defined. It can be seen that the larger the PD(*q*), the larger the *H*(*q*), and then, the higher the strength of privacy protection [29].

The article "Clinical Analysis of the Renal Protective Effect of GLP-1 on Diabetic Patients Based on Edge Detection" was published in 2022. Journal: J Healthc Eng.

After obtaining the privacy metric, the privacy risk of information leakage in complex environments can be assessed by performing various rich heterogeneous information deanonymization attacks on various existing information amortization methods, or by designing new edge computing-based attacks in a targeted manner to obtain the privacy metric of different information amortization methods in the face of different attacks, and then give a statistically significant quantitative index of privacy leakage risk.

For the needs of different service functions, data is classified and operated, combined with function encryption (e.g., attribute-based encryption) methods, and fine-grained access control schemes are developed for the sharing and use of data in collaboration with the computing and storage resources of terminal devices and edge devices. First, data generated by user terminals are classified, such as user personal information *M*_0_ and data for different service functions (*M*_0_, ⋯, *M*_*n*_), according to different security requirements. In general, the user's personal information only needs to be accessed by the service provider when personalised services are provided to the user, but service information can provide the basis for global resource analysis.

As a result, users' personal information requires a stronger protection scheme than service information. In order to achieve fine-grained access control, users can store personalised information on local terminals and submit service information to edge and cloud servers for analysis and management. Furthermore, it is also possible to implement a more granular management of data for different functions.

## 4. Case Studies

### 4.1. Source

Eighty patients with DKD were admitted to our hospital meeting the criteria for DKD diagnosis, signing the informed consent form. Exclusion criteria are as follows: age <18 years; allergic to study drugs; patients on dialysis; patients with serious cardiovascular, gastrointestinal, respiratory, neurological or endocrine diseases; patients with major surgery or severe trauma; pregnant or lactating women; patients with combined diabetic ketoacidosis, acute and chronic infections, malignant tumours, etc.; patients with poor adherence and unable to take medication regularly; patients with poor compliance or inability to take medication regularly; and other patients who, in the opinion of the investigator, are not suitable for participation in the study. The study was approved by the hospital ethics committee and all patients gave their informed consent. 80 patients included were randomly divided into observation and control groups according to a random number table, with 40 patients in each group. Clinical data such as age, sex, body mass index, and duration of diabetes were compared and analysed between the two groups.

The article "Clinical Analysis of the Renal Protective Effect of GLP-1 on Diabetic Patients Based on Edge Detection" was published in 2022. Journal: J Healthc Eng.

Fasting peripheral venous blood was collected from the patients in the morning in a normal blood collection tube, left to stand at room temperature until the blood was completely clotted, centrifuged, and the serum was separated. The fasting blood glucose (FBG) level was measured by the glucose oxidase method, and the glaciated haemoglobin (HbA1c) level was measured by high-performance liquid chromatography. Continuous glucose monitoring system (CGMS) was used to monitor all patients' ambulatory blood glucose levels, and the 24 h mean blood glucose (MBG), standard deviation of blood glucose (SDBG), and blood glucose levels were measured. Glucose (SDBG), 24 h blood glucose fluctuation range (BGFR), and mean amplitude of glyce-mic excursions (MAGE) are monitored [30].

### 4.2. Results

There were no statistically significant differences in clinical data such as age, gender, body mass index, and duration of diabetes between the two groups (*P* > 0.05) [31–33].  Table 1 is comparison of clinical information between the two groups of patients.

After 24 weeks of treatment, FBG, HbAlc, MBG, SDBG, BGFR, and MAGE were significantly lower in both groups than before treatment (*P* < 0.05). The differences in FBG, HbAlc, MBG, SDBG, BGFR, and MAGE between the two groups before treatment were not statistically significant (*P* > 0.05).

The differences in Scr, Umalb, and ACR between the two groups before treatment were not statistically significant (*P* > 0.05); at 24 weeks of treatment, Scr, Umalb, and ACR were significantly lower in both groups than before treatment (*P* < 0.05), and Scr, Umalb, and ACR were significantly lower in the observation group than in the control group (*P* < 0.05); at 24 weeks of treatment, the eGFR of patients in the observation group was significantly higher than that before treatment (*P* < 0.05), and the eGFR of patients in the observation group was significantly higher than that of the control group (*P* < 0.05).

At 24 weeks of treatment, serum AGEs and cAMP levels in the control group were significantly lower than those before treatment (*P* < 0.05), while the differences in serum MDA, SOD, and CAT levels before and after treatment were not statistically significant (*P* > 0.05); serum AGEs are low before treatment (*P* < 0.05), while serum SOD and CAT levels were significantly higher than those before treatment (*P* < 0.05). The serum AGEs, cAMP, and MDA in the observation group were significantly lower (*P* < 0.05), while the serum SOD and CAT levels were significantly higher (*P* < 0.05).

The article "Clinical Analysis of the Renal Protective Effect of GLP-1 on Diabetic Patients Based on Edge Detection" was published in 2022. Journal: J Healthc Eng.

The levels of PKA and p-CREB in peripheral blood mononuclear cells in the observation group were significant, but the difference in CREB protein levels was not statistically significant (*P* > 0.05). The differences in the levels of PKA, CREB, and p-CREB in peripheral blood mononuclear cells between the two groups before treatment were not statistically significant (*P* > 0.05), while the levels of PKA and p-CREB in peripheral blood mononuclear cells in the observation group at 24 weeks of treatment were significantly lower than those in the control group (*P* < 0.05), but the levels of CREB protein levels were not statistically significant compared with the control group (*P* > 0.05) [34–36].  Figure 4 displays measurement of PKA/CREB signalling pathway-related proteins in peripheral blood mononuclear cells before and after treatment in two groups of patients.

In metabolic syndrome, the body's regulation of adiposity is disturbed, leading to a disturbance in lipid metabolism. The present study confirmed that TNF-*α* expression was upregulated in patients with diabetes and diabetic combined metabolic syndrome, with more pronounced upregulation in patients with diabetic combined metabolic syndrome, suggesting that the patients were in an inflammatory state. TC, waist circumference, TNF-*α*, TG, systolic blood pressure, diastolic blood pressure, GHb, and fasting glucose were negatively correlated with GLP-1 expression. It is suggested that monitoring the abovementioned indicators can help predict the progression of type 2 diabetes and the development of metabolic syndrome, which is a guideline for the diagnosis and treatment of the disease.

DKD is characterized by the accumulation of extracellular matrix in the glomerular mesenchyme and tubulointerstitial matrix, leading to thickening of the glomerular basement membrane, thylakoid hyperplasia, tubulointerstitial fibrosis, and ultimately irreversible renal fibrosis. The main pathogenic mechanisms include disturbances in glycolysis metabolism, oxidative stress, activation of inflammatory signalling pathways, altered haemodynamics, nonenzymatic generation of proteins, activation of polymer pathways, and activation of the renin-angiotensin II-aldosterone system (RAS), with the involvement of a variety of different cells and cytokines. However, the specific molecular mechanisms of action remain elusive. There is a lack of effective treatment for DKD, and the main clinical approach is to control blood pressure and blood glucose and reduce protein intake, but the improvement of proteinuria that has already occurred is limited.  Figure 5 presents diabetes clustering for different edge computing.

The article "Clinical Analysis of the Renal Protective Effect of GLP-1 on Diabetic Patients Based on Edge Detection" was published in 2022. Journal: J Healthc Eng.

Glucagon-lipopeptide-1 (GLP-1) has been one of the hot topics of research in diabetes treatment in recent years. Exempted is the first GLP-1 agonist approved for clinical use, lowering blood glucose in a glucose-dependent manner, rarely causing hypoglycaemia when used alone, reducing body mass and improving lipid metabolism and islet function in patients with type 2 diabetes mellitus (T2DM) patients, improving lipid metabolism and islet function. As shown in Figure 6, the calculated efficiencies of GLP-1 at different nodes indicate that, in addition to hypoglycaemic effects, GLP-1 is also a multidrug agent with antioxidative stress and inhibition of apoptosis and has been shown to have a protective effect on the kidney in diabetes. In this study, we investigated the renal protective effect of exempting in DKD patients and its mechanism of action. Figure 6 is computational efficiency of different algorithms for different nodes.

## 5. Conclusions

Under the background of global interconnection and interconnection of all things, intelligent medical treatment is the ultimate goal of realizing medical informatization. At the same time, considering the disadvantages of cloud computing. It has gradually failed to meet the timeliness of intelligent medical treatment for big data processing and information interaction. Therefore, the combination of intelligent medical treatment and edge computing is the requirement of the time. This paper introduces the related technologies of smart medical combined with edge computing and the security and privacy problems it faces. At the same time, for this problem, referring to the solutions proposed in some parts, this paper puts forward its own private security protection framework and some solutions. Safe operation is an important guarantee for the growth of smart medical under the edge computing system. Therefore, ensuring the privacy and security of intelligent medical edge computing system is the booster to make medical informatization intelligent.

## Figures and Tables

**Figure 1:** Edge computing architecture for smart healthcare.

**Figure 2:** Sources of privacy and security concerns.

**Figure 3:** Core framework for research on privacy security protection.

**Figure 4:** Measurement of PKA/CREB signalling pathway-related proteins in peripheral blood mononuclear cells before and after treatment in two groups of patients.

**Figure 5:** Diabetes clustering for different edge computing.

The article "Clinical Analysis of the Renal Protective Effect of GLP-1 on Diabetic Patients Based on Edge Detection" was published in 2022. Journal: J Healthc Eng.

**Figure 6:** Computational efficiency of different algorithms for different nodes.

**Table 1:** Comparison of clinical information between the two groups of patients.

Group	Age (years)	Gender (*n* (%))		Body mass index (kg/m^2^)	Diabetes course (year)
		Male	Female sex		
Control group	56.42±11.85	24	16	26.67±2.73	9.47±3.56
Observation group	55.68±12.21	22	18	27.39±2.81	8.95±4.17
*t*/*x*^2^ value	0.275	0.205	1.162	0.6	
*P* value	0.785	0.651	0.252	0.552	

## Data Availability

The data used to support the findings of this study are available from the author upon request.
